The article "TMED3 promotes cell proliferation and motility in breast cancer and is negatively modulated by miR-188-3p" was retracted in 2024. Reasons: duplicated images; overlap with earlier publications; unreliable results or conclusions; concerns about the results or conclusions.

# TMED3 promotes cell proliferation and motility in breast cancer and is negatively modulated by miR-188-3p

**DOI:** 10.1186/s12935-019-0791-4

**Published:** 2019-03-29

**Authors:** Jing Pei, Jing Zhang, Xiaowei Yang, Zhengsheng Wu, Chenyun Sun, Zhaorui Wang, Benzhong Wang

**Affiliations:** 1 Department of Breast Surgery, Department of General Surgery, The First Affiliated Hospital of Anhui Medical University, Number 218, Jixi Road, Hefei, 230022 Anhui People’s Republic of China; 2 Department of Breast Surgery, The Tumor Hospital of XuZhou, HuanCheng Road 131, Xuzhou, 221003 Jiangsu People’s Republic of China; 3 Department of Pathology, The First Affiliated Hospital of Anhui Medical University, Jixi Road 218, Hefei, 230022 Anhui People’s Republic of China

**Keywords:** Breast cancer, TMED3, miR-188-3p, Prognosis, Migration

## Abstract

**Background:**

The role of TMED3 involved in cancers has been seldom described, let alone in breast cancer. To explore the clinicopathological significance of TMED3 expression and the biological roles involved in breast cancer cells, we undertook the study.

**Methods:**

Immunohistochemistry was performed to observe the pattern of TMED3 expression in breast cancer tissues, totaling 224 cases; followed by detailed statistical analysis between TMED3 expression versus clinicopathological information available. To explore the role of TMED3 involved in the malignant behaviors of breast cancer cells, wound-healing and Transwell assays were conducted to evaluate the variation of migration and invasion of MCF-7 and MDA-MB-231 cells whose TMED3 has been stably silenced using lenti-viral based short hairpin RNA (shRNA) vectors. MTT, clonogenic assay and xenograft nude mice model were undertaken to observe the variation of proliferation both in vitro and in vivo.

**Results:**

It was shown that elevated TMED3 markedly correlated with ER, PR, Her-2 status, and lymph nodes metastases in addition to significant association with poor overall prognosis. In vitro, TMED3 was shown to promote proliferation, migration and invasion of breast cancer cells. Moreover, miR-188-3p was identified as a novel negative regulator of TMED3 in breast cancer, which can slow down the proliferation, migration and invasion of MCF-7 cells. Results from in vivo xenograft nude mice models showed that lenti-viral based miR-188-3p re-expression can markedly impair the tumor growth.

**Conclusions:**

Our data define and bolster the oncogenic role of TMED3 in breast cancer.

**Electronic supplementary material:**

The online version of this article (10.1186/s12935-019-0791-4) contains supplementary material, which is available to authorized users.

## Background

Breast cancer is one of the most common types of cancer diagnosed among women world-wide and the second leading cause of cancer death among women in the US [1]. In China, the burden of female breast cancer is getting increasingly severe, especially in urban areas of China [2]. Despite the great advancement in the understanding, surgical and meditations; breast cancer remains to be a major cause of death worldwide [3]. Consequently, further investigation of novel oncogenes involved in the pathogenesis of breast cancer is needed and necessary.

TMED3, a contraction of Transmembrane Emp24 Protein Transport Domain Containing 3, a member of TMED family thought of being implicated in the vesicular trafficking of proteins and innate immune signaling [4]. Till now, the ten members of TMED family have been discovered [5]; many TMED proteins [6–9] have been investigated and reported except for TMED3 which has been comparatively seldom described in the context of cancer, with the exception of the only three relevant studies performed regarding TMED3 in cancers, including prostate cancer [10], colon cancer [11] and liver cancer [12]. Evidence from the three studies of TMED3 suggest the role of TMED3 involved in malignancies seems to be different even somewhat controversial. Considering that no evidence has been available concerning TMED3 in breast cancer, herein we attempted to explore both of the clinicopathological and biological roles of TMED3 in breast cancer. We firstly defined the oncogenic role of TMED3 in breast.

## Methods

### Tissue microarray preparation

Formalin-fixed, paraffin-embedded blocks of breast cancer and its paired normal control tissues, totaling 224, were retrieved from the archives at the Department of pathology, The First Affiliated Hospital of Anhui Medical University. All these blocks we retrieved were outsourced to prepare the tissue microarray by Shanghai Outdo Biotech Co. Ltd. (Shanghai, China). Another additional independent 37 cases of fresh frozen breast cancer tissues were collected in The Department of Breast Surgery, The First Affiliated Hospital of Anhui Medical University. All cancer tissues were staged and graded following the World Health Organization classification and grading system (2016 version). None of the patients had received any treatment before mastectomy. Both the cancer and its adjacent normal controls were histopathologically confirmed by experienced pathologist (Zhengsheng Wu M.D) who was totally blind to our study from the outset. Informed consent was obtained from each participant involved, and the study got approval from the Medical Ethics Committee of the First Affiliated Hospital of Anhui Medical University.

### Cell culture and siRNA transfection

The human breast cancer cell lines MDA-MB-231, MDA-MB-468 and MCF-7 as well as the normal human breast mammary epithelial cell lines MCF-10A were commercially from American Type Culture Collection (ATCC, Manassas, VA, USA). The transformed but not malignant human mammary epithelial cell line HBL-100 (HBT-124, ATCC, USA) has been routinely stored in liquid nitrogen in our cell laboratory in The First Affiliated Hospital of Anhui Medical University. The MCF10A cells were cultured in a DMEM/F12 medium containing EGF (20 ng/mL), hydrocortisone (0.5 mg/mL), cholera toxin (100 ng/mL) (Sigma-Aldrich; St. Louis, MO, USA), insulin (10 μg/mL), and 1× penicillin–streptomycin (Gibco; Carlsbad, CA, USA). HBL-100 cell line was cultured in MEM media supplemented with 10% fetal calf serum, 0.2% sodium bicarbonate, 10 mM HEPES, 1% non-essential amino acids, 2 mM l-glutamine and 6 ng/mL insulin (Life Technologies, Grand Island, NY USA). The breast cancer cells were cultured in DMEM (HyClone; Logan, UT, USA) supplemented with 10% fetal bovine serum (FBS; Gibco). All cells were maintained at 37 °C in a humidified 5% CO_2_ atmosphere incubator. The specific siRNA to TMED3 was designed and synthesized by GenePharm Company (GenePharma, Shanghai, China), the sequences were tabulated in Additional file 1: Table S1. The lenti-viral based shRNA for TMED or re-expression of miR-188-3p vectors were outsourced to GeneChem Company (GeneChem, Shanghai, China) to construct. Cells were seeded in six-well plates at the concentration of 4 × 10^5^ cells/well 24 h before the transfection with TMED3-siRNA and its control using Lipofectamine™ 2000 (Invitrogen, Life Technologies Inc, USA) following the manufacturer’s instructions.

### Quantitative real-time PCR (qRT-PCR)

Total RNA were isolated using the Trizol (Invitrogen™, Life Technologies Inc, USA) according to the manufacture’s protocol. RNA from each sample was transcribed into cDNA using Revert Aid First Strand cDNA Synthesis Kit (Catalog number: K1621, Thermo Fisher Scientific, MA, USA) according to the manufacturer’s instructions. qRT-PCR was conducted using Fast Start Universal SYBR Green Master (Rox) (Roche, Germany). TMED3 PCR detection was performed using SYBR Green method (Catalog number: 4309155, Thermo Fisher Scientific, MA, USA). The PCR cycle consisted of 95 °C for 3 min, 95 °C for 30 s, 62 °C for 30 s (β-actin was 55 °C for 30 s), 72 °C for 30 s. Expression of TMED3 was normalized to the β-actin to control the variability in expression levels. The relative expression levels were calculated using standard curve method. The sequence of primers was listed in Additional file 1: Table S1.

### Immunohistochemistry (IHC)

The tissue microarray was incubated at 60 °C overnight and then subjected to de-paraffinization and dehydration in gradient ethanol. The activity of endogenous peroxide was blocked in 3% H_2_O_2_ for 15 min. The antigen was retrieved in 0.01 M citrate buffer heated in a microwave oven at 98 °C for 15 min and then was cooled at room temperature for 15 min. After washing in phosphate-buffered saline (PBS), the tissue microarray was incubated with normal serum to block nonspecific staining for 30 min. Polyclonal rabbit anti-TMED3 (1:150 dilution; Ab151056, Abcam, MA, Cambridge, USA) was incubated with the tissue section overnight at 4 °C in a humidified chamber. After washing with PBS, the tissue section was treated with biotinylated anti-mouse secondary antibody, followed by further incubation with streptavidin–horseradish peroxidase complex and staining using the diaminobenzidine kit (Beijing Zhongshan Golden Bridge Biotechnology Co, Ltd). IHC staining was assessed in a series of randomly selected four fields at 400× magnification.

### Immunoscoring of TMED3

Four fields per section were randomly selected, and the immunostaining of TMED3 was scored by two separate clinical pathologists. The immunostaining of TMED3 was classified into the following four categories: 0, negative (no positive cells); 1, weak positive (between 20% and 40% positive cells per mm^2^); 2, moderate positive (between 40% and 60% positive cells per mm^2^); 3, strong positive (> 60% per mm^2^). For statistical analysis, these categories were categorized into two groups, low (0–1) and high (2–3) expression.

### Flow cytometry analysis

Cells were harvested with tyrosine after transfection for 48 h, fixed with cold 70% ethanol at 4 °C overnight, followed by adding RNase A enzyme (0.05 mg/mL) and staining with propidium iodide (PI, 0.05 mg/mL), cell cycle distribution was analyzed on a FACS Calibur system (3550UV, BioRad, USA). For apoptosis detection, cells were stained by the Annexin V-FITC kit (Invitrogen™, Life Technologies Inc, USA) following the accompanying instruction. Viable cells were not stained with Annexin V. The necrotic cells were Annexin V and PI double positive, whereas apoptotic cells were Annexin V positive and PI negative.

### Mitomycin C treatment

Cells were trypsinized (0.25% trypsin–EDTA; Invitrogen™, Life Technologies Inc, USA) for 2 min at 37 °C, washed with SMC medium, and then incubated as a single-cell suspension in 40 μg/mL Mitomycin-C (catalog number: M4287; Sigma-Aldrich Chemical Company, St. Louis, MO, USA) in DMEM medium for 30 min at 37 °C. After two additional washes in PBS, cells were assessed for viability, proliferation, or migratory ability. For the wound healing assay, Mitomycin-C treatment was performed after DMEM plating and when cells were 100% confluent; cells were incubated in 40 μg/mL mitomycin-C in DMEM medium for 30 min at 37 °C and then washed twice in PBS before assay.

### MTT

Cells were placed in a 96-well plate at a density of 4 × 10^3^/well and were incubated overnight. At 0, 24, 48, 72, and 96 h, 20 μL (5 g/L) of MTT (3-(4,5-dimethyl-2-thiazolyl)-2,5-diphenyl-2-*H*-tetrazolium bromide) reagent was added to the designated wells. After a 4 h incubation, the MTT formazan precipitate was dissolved in dimethylsulphoxide (DMSO) (150 μL/well, Sigma-Aldrich, St. Louis, MO, USA) in a shaker before reading the absorbance at 490 nm using a 96-well plate reader (Bio-Rad, Winooski, VT USA).

### Wound healing assay

Cells were seeded in 6-well plates. After overnight incubation, the cells were preceded by treatment with Mitomycin C (40 μg/mL) for 30 min; followed by scrape with a 10 µL pipette tip to generate a straight-line cell-free scratch. Migrating cells were photographed after 24 h. Each well was washed with PBS to remove the remaining unattached cells before imaging. Cell motility was quantified by measuring the distance between the migrating cell boundaries.

### Transwell assay

Transwell assay was performed to assay the invasion and migration of breast cancer cells using a 24-well Transwell chamber with a polycarbonate membrane with a pore size of 8 μm (Corning, NY, USA). The membrane was coated with or without 60 μL of a 1:5 mixture of Matrigel (BD Sciences, San Jose, CA, USA) and serum-free DMEM medium to form a matrix barrier. After the Matrigel was allowed to solidify at 37 °C for 2 h, breast cancer cells (1 × 10^5^ cells/mL) were pretreated with Mitomycin C (40 μg/mL) in 200 µL of serum-free DMEM medium were added to the upper compartment of the chamber; The lower chamber was filled with 0.6 ml of medium supplemented with 10% FBS as a chemo-attractant. After incubation at 37 °C for 24 h, cells were then rinsed with PBS and fixed in 100% methanol. The cells remaining at the top of the polycarbonate membrane were removed using a moist cotton-tipped swab. The cells that migrated through pores to the lower surface were stained with crystal violet and hematoxylin and distilled water several times, and the cell numbers in four random fields at a magnification of 200× were counted and averaged.

### Clonogenesis assay

Clonogenic growth of breast cancer cells were assessed by incubating 500 cells transfected with lentiviral-based shTMED3 or re-expression of miR-188-3p vectors that were preceded by previously cell sorting for GFP expression using Flow Cytometry. Clonogenic cultures were performed in 12-well plate in 1 ml in DMEM (HyClone; Logan, UT, USA) supplemented with 10% fetal bovine serum (FBS; Gibco). Colonies of more than 50 cells were automatically counted using Image J software (NIH, Bethesda, MA, USA) after 10 days.

### miRNA target prediction and luciferase reporter assay

The potential targets of miR-188-3p were predicted using miRanda (www.microrna.org) and TargetScan (www.targetscan.org). TMED3 was found to be a putative target of miR-188-3p. The 3′-UTR of TMED3 containing the complementary sequences of miR-188-3p or mutation sequences was amplified and subcloned into the pMirTarget plasmid (Origene, Rockville, MD, USA), which were named as pMirTarget-TMED3-3′-UTR wild-type (WT) and pMirTarget-TMED3-3′-UTR mutant (MUT), respectively. Cells were inoculated into 24-well plates 1 day before transfection. Cells were co-transfected with miR-188-3p mimics or miR-NC, and pMirTarget-TMED3-3′-UTR WT or MUT, using Lipofectamine 2000^®^. Following 48 h of incubation at 37 °C, the luciferase activity was determined using a Dual-Luciferase Reporter Assay system (Promega Corporation, Madison, WI, USA). Renilla luciferase activity was chosen for normalization.

### Western blot

Cells were lysed in RIPA lysis buffer. The protein concentrations were determined using the BCA protein quantitation assay (Bioteke, Beijing, China). Equal amounts of protein (50 μg) were separated on 12% SDS-PAGE gels and were transferred to a PVDF membrane (Millipore, Bedford, MA, USA). The membranes were blocked for 1 h using blocking buffer and then were probed overnight with an anti- TMED3 Rabbit mAb (1:800; ab173112, Abcam, MA, Cambridge, USA), and anti-GAPDH antibody (1:1000; #5174; Clonality: D16H11; Cell Signaling Technology) at 4 °C. The membrane was washed three times for 5 min each time with washing buffer and was incubated with secondary antibody anti-rabbit IgG, Fluorescence-linked antibody (catalog number: 926-32211; LI-COR Biosciences, Lincoln, Nebraska, USA) dilution at 1:10,000, incubation for 1.5 h avoid light at 37 °C. Proteins were detected using LI-COR Odyssey Imaging system (LI-COR Biosciences, Lincoln, Nebraska, USA).

### Xenograft nude mice model

All animal procedures were carried out following the procedures described in the Laboratory Animal Maintenance Manual of The First Affiliated Hospital of Anhui Medical University (Approval No. AHMU-F1-111208). Six-week-old male nude mice (BALB/cSlcn/n) were purchased from Vitalriver Inc. (Vitalriver, Beijing, China) and maintained under specific pathogen-free conditions. For subcutaneous implantation, tumors were established by injecting MCF-7 cells expressing either control or pcDNA6-miR-188-3p at the density of 1 × 10^7^ cells subcutaneously into the left flank of each mouse. Mice were divided into six groups and tumor lesions were harvested 1 month later.

### Statistical analysis

The data were expressed as the mean ± standard error of mean (SEM). Statistical analysis was carried out using SPSS 17.0 software (SPSS, Chicago, IL, USA). Independent sample T-test and one-way ANOVA were used for statistical analyses between groups of continuous variables that followed the normal distribution. Cross-table analysis was conducted for categorical variables. Kaplan–Meier survival analysis was performed for overall prognostic analyses. A value of p < 0.05 was taken as statistically significant.

## Results

### Up-regulated TMED3 remarkably correlated with poor overall survival in breast cancer

To learn about the expression pattern of TMED3 in breast cancer tissues, immunohistochemistry (IHC) was carried out on tissue microarray consisting of 112 cases breast cancer tissue dots. IHC detection revealed the highly heterogenous expression of TMED3, with the immunostaining varying from case to case from being negative, weak, and moderate to strong positive in breast cancer tissues (Fig. 1a–d). By contrast, TMED3 was hardly detectable or weak positive immunostaining of TMED3 predominates in paired normal controls (Fig. 1e, f). Taken as a whole, TMED3 was shown to be pronouncedly up-regulated in breast cancer tissues compared with its matched normal controls (Table 1). Subsequent statistical analysis with clinicopathological variables, including overall survival, age, estrogen receptor (ER), progesterone receptor (PR), human epidermal growth factor receptor-2 (Her-2), M classification, N classification, subtyping, grading and staging. It exhibited that up-regulated TMED3 was markedly associated with inferior overall prognosis (Fig. 1g). Moreover, TMED3 remarkably correlated with ER, PR, Her-2, and lymph nodes metastases. No significant correlation was observed between TMED3 expression and other pathological variables, including age, M classification, subtyping, grading and staging. As complement, qRT-PCR was conducted on mRNA level with fresh frozen breast cancer tissues, totaling 37 cases. Consistently, results from qRT-PCR presented that TMED3 mRNA was remarkably elevated in breast cancer tissues as compared with normal control (Fig. 1h). In addition, western-blot was also carried out to confirm TMED3 expression on limited 10 paired cases of fresh breast cancer and its normal controls. The results of western-blot exhibits that compared with normal control, TMED3 was displayed to be markedly over-expressed in breast cancer tissues (Fig. 1). Together, all the data we collected demonstrated that elevated TMED3 in breast cancer was significantly associated with poor overall survival (Table 2).

**Fig. 1:** Up-regulated TMED3 significantly is associated with unfavorable overall prognosis in breast cancer. **a** Strong immunostaining of TMED3; **b** moderate staining of TMED3; **c** weak staining of TMED3; **d** negative staining of TMED3 in breast cancer tissue; **e** negative staining of TMED3 in normal breast tissue; **f** moderate staining of TMED3 in the duct of normal breast tissue. Scale bar stands for 5 µm; magnification fold for overview of dots was ×5, whereas ×40 for insets. Shown were the representative figures selected from candidates. **g** Kaplan–Meier survival curve of TMED3 expression in patients with breast cancer, divided into high and low group according to the status of TMED3 expression, with each group having 59 and 53 cases respectively. Log-rank test was used to analyze the difference of overall survival. **h** qRT-PCR detection of TMED3 expression on mRNA level in 37 cases of breast cancer and its matched normal control tissues. ***p < 0.001 compared with control normal group using independent sample T-test; **i** western-blot analysis of TMED3 in the fresh breast cancer tissues, totaling 10 paired cases. *T* tumor tissue, *N* normal breast tissue. The molecular weight (MW) of TMED3 was around 25 kDa, β-actin, as internal loading control whose MW was observed to be about 42 kDa. Quantitative assay was performed using Image J software (NIH, Bethesda, USA), ***p < 0.001 relative to control group using independent sample T-test

**Table 1:** Clinicopathological significance of TMED3 expression in breast cancer

Characteristics	N	TMED3 expression		χ^2^	*p*
		Low	High		
Breast cancer	112	53	59	45.551	0.000
Matched normal	112	100	12		
Age (years)					
< 50	49	24	25	0.096	0.849
≥ 50	63	29	34		
Tumor size (cm)					
≤ 2	38	17	21	0.154	0.842
> 2	74	36	38		
ER					
+	85	41	44	8.703	0.003
−	27	11	16		
PR					
+	54	38	16	3.386	0.050
−	58	31	27		
Her-2					
+	50	23	27	4.579	0.037
−	62	41	21		
M classification					
M0	78	38	40	0.201	0.685
M1–3	34	15	19		
N classification					
N0	51	14	37	14.831	0.000
N1–3	61	39	22		
Subtype					
Luminal A	15	7	8	0.042	1.000
Luminal B	56	27	29		
Her-2	17	8	9		
Triple-negative	24	11	13		
Grading					
I	21	12	9	3.492	0.181
II	55	29	31		
III	36	12	24		
Staging					
I + II	67	37	30	4.177	0.054
III + IV	45	16	29

**Table 2:** Univariate analysis and multivariate analysis for predictors of overall survival

Variables	Univariate analysis			Multivariate analysis		
	HR	CI	*p*	HR	CI	*p*
Age	1.782	1.077–2.947	0.024	1.637	0.769–3.483	0.303
Tumor size	0.389	0.177–0.855	0.019	1.404	0.762–2.587	0.245
N classification	0.160	0.079–0.324	0.000*	0.192	0.092–0.400	0.000*
Grading	0.554	0.287–1.271	0.184	0.757	0.347–1.652	0.484
ER status	0.413	0.187–0.540	0.000*	0.345	0.155–0.768	0.496
PR status	0.457	0.270–0.737	0.002	1.302	0.609–2.783	0.006
HER-2 status	1.013	0.615–1.287	0.018	1.914	1.253–3.724	0.021
Staging	1.422	1.379–3.185	0.068	1.687	0.914–2.849	0.083
TMED3	3.059	1.763–5.309	0.000*	1.852	1.013–3.387	0.017

Variables: age, > 48 vs. ≤ 48; tumor size, < 2 cm vs. ≥ 2 cm, LNM, negative vs. positive, Chemotherapy, yes vs. no; ER status, positive vs. negative; PR status, positive vs. negative; HER-2 status, positive vs. negative; Ki-67 status, positive vs. negative; TMED3, high expression vs. low expression; Cox proportional hazards model; “*” represent “p < 0.001”

*HR* hazard ratio, *CI* confidence interval, *TMED3* transmembrane P24 trafficking protein 3, *ER* estrogen receptor, PR progesterone receptor, *HER-2* human epidermal growth factor receptor-2, *Ki-67* protein encoded by the MKI67 gene

### TMED3 promotes proliferation and motility of breast cancer cells

Having seen the expression pattern of TMED3 in breast cancer tissues, next we explored the biological roles of TMED3 involved in the proliferation and motility of breast cancer cells. First of all, four different kinds of cell lines were enrolled, including two kinds of breast cancer cell lines MDA-MB-231 and MCF-7 and two kinds of control cell lines HBL-100 and MCF-10A. Basal level of TMED3 was determined using western-blot, showing that TMED3 was remarkably higher in MDA-MB-231 and MCF-7 cell lines than that in control cell lines (Fig. 2a). Yet, little significant difference of TMED3 was observed between MDA-MB-231 and MCF-7 cell line. Here, TMED2 and TMED4, two important paralogs of TMED3 from the same super family, have to be mentioned here. We also wonder the expression status of TMED2 and TMED4 while detecting the TMED3 expression; thus, the detection of TMED3 was extended to TMED2 and TMED4 in different breast cancer cell lines (Additional Figure S1A). It showed that both of TMED2 and TMED4 can be detected in MCF-7 and MDA-MB-231 cells (Additional file 1: Figure S1B, C). Next, small interference RNAs (siRNAs) to human TMED3 at three different sites of TMED3 mRNA, termed TMED3-siRNA-1, TMED3-siRNA-2, and TMED3-siRNA-3 respectively, were used and transfected, followed by evaluation of the silencing effect of these siRNAs in MCF-7 and MDA-MB-231 cells. It can be seen that among the three siRNAs that can all work, the knock-down effect of siRNA named TMED3-siRNA-1 was most significant of all (Fig. 2b, c). Consequently, TMED3-siRNA-1 was selected to further construct the lenti-viral based short-hairpin RNA (shRNA) vector. As expected, shRNA-TMED3 (hereafter referred to as sh-TMED3) can stably and effectively knock down TMED3 in MCF-7 and MDA-MB-231 cells (Fig. 2d). Based on which, we subsequently assessed the variation of proliferation, migration and invasion in MCF-7 and MDA-MB-231 cells where TMED3 was stably knocked down. MTT assay showed that knock-down of TMED can drastically impair the proliferation in MCF-7 and MDA-MB-231 cells (Fig. 3a, b), which was corroborated by clonogenic assay performed in MCF-7 and MDA-MB-231 cells (Fig. 3c, d). To exclude the potentially confounding influence that may be caused by proliferation in the analysis of migration and invasion, all breast cancer cells underwent pretreatment with Mitomycin C to eliminate the proliferative influence before undergoing the wound-healing and Transwell assays. Wound-healing assay exhibited that migratory abilities were significantly suppressed after TMED3 was being stably silenced in MCF-7 and MDA-MB-231 cells (Fig. 3e, f). Likewise, the invasive abilities were also pronouncedly abrogated after TMED3 was being silenced, as exemplified by Transwell assay performed in MCF-7 and MDA-MB-231 cells (Fig. 3g, h). Moreover, the variation of both the apoptosis and cell cycle after silencing of TMED3 was also incidentally analyzed using Flow Cytometry. It showed that silencing of TMED3 can dramatically induce the apoptosis in breast cancer cells through decreasing the S phase (Additional file 1: Figure S2). Together, the data strongly suggests that TMED3 can promote the proliferation, migration and invasion of breast cancer cells.

**Fig. 2:** TMED3 was expectedly elevated in breast cancer cell lines. **a** Basal expression of TMED3 in breast cancer cell lines MDA-MB-231 and MCF-7 as well as the normal human breast mammary epithelial cell line MCF-10A and the transformed but not malignant human mammary epithelial cell line HBL-100, as detected by western-blot; **b** silencing effect of siRNA sequences targeting TMED3 was evaluated by western-blot in MCF-7 cell line; **c** likewise, the transient knock-down efficiency was evaluated in parallel in MDA-MB-231 cell line; **d** stable knock-down efficiency of lenti-viral based short hairpin RNA (shRNA) targeting TMED was detected using western-blot in both MCF-7 and MDA-MB-231 cell lines. All detections were done independently three times and shown were the representative figures selected among candidates. Quantitative analysis was carried out using Image J software (NIH, Bethesda, USA)

**Fig. 3:** TMED3 promotes proliferation, migration and invasion in breast cancer cell lines. **a**, **b** Stable knock-down of TMED3 was shown to markedly impair the proliferation in MCF-7 and MDA-MB-231 cell lines, as exemplified by MTT assays; **p < 0.01, ***p < 0.001 in comparison with control group using independent sample T-test method; **c**, **d** clonogenic abilities were shown to be remarkably suppressed after TMED was being stably silenced in MCF-7 and MDA-MB-231 cell lines, as detected by clonogenesis. **p < 0.01, ***p < 0.001 compared with control group using independent sample T-test; **e**, **f** migration was significantly slowed down after TMED being stably knocked down in MCF-7 and MDA-MB-231 cell lines, as detected by wound-healing assays. **p < 0.01 relative to control group using independent sample T-test; **g**, **h** similarly, invasion was also inhibited when TMED3 was stably silenced in MCF-7 and MDA-MB-231 cell lines, as evaluated by Transwell assays.*p < 0.05, **p < 0.01 compared with control group using independent sample T-test. All experiments were performed independently three times and presented were the representative figures among candidates

### MiR-188-3p was identified as negative regulator of TMED3

Inspired by the miRNA-mRNA modulation mode, we next attempted to screen out the potential miRNAs that can regulate the TMED3 using miRNA microarray platform. It showed that there were as many as five different miRNAs that were screened out to be indicative of potential regulators of TMED3 (Fig. 4a). Having reviewed the relevant literatures regarding the five miRNAs we obtained, we picked out the miR-188-3p as miRNA of interest to further confirm. Meanwhile, bioinformatic analysis using Targetscan software on-line theoretically predicted that there were two potential binding sites in the 3′-untranslated region (3′-UTR) of TMED3 (Fig. 4b and Additional file 1: Figure S3). As further confirmation, luciferase reporter assay was performed exhibiting that miR-188-3p can bind the 3′-UTR of TMED3, regardless of breast cancer cell lines used (Fig. 4c, d). Subsequently, to understand the regulation exerted bymiR-188-3p over TMED3, variation of mRNA of TMED3 was detected using qRT-PCR technique after forced or abrogated expression of miR-188-3p. It was observed that TMED3 mRNA was drastically decreased with forced expression of miR-188-3p, whereas mRNA of TMED3 rebounded significantly with inhibition of miR-188-3p, strongly suggesting the negative regulation of miR-188-3p on TMED3 (Fig. 4e), which was fully corroborated by western-blot analysis of variation of TMED3 in MCF-7 and MDA-MB-231 cells on protein level (Fig. 4f, g). Additionally, expression level of miR-188-3p was detected using qRT-PCR in 37 paired cases of breast cancer and its matched normal controls. MiR-188-3p was displayed to be markedly lower in breast cancer tissues compared with normal controls (Fig. 4h). The correlation between mRNA of miR-188-3p and TMED3, by Pearson Correlation analysis, verifies the negative correlation between them on tissue level (Fig. 4i). All the data we gleaned demonstrates that miR-188-3p can negatively regulate the TMED3, playing an anti-oncogenic role in breast cancer.

**Fig. 4:** TMED3 was identified as a down-stream target of miR-188-3p. **a** Most significantly up-regulated miRNAs, totaling 5, were screened out using miRNA microarray analysis between group transfected with si-TMED3 and control group, with each group in triplicate. **b** Conservation of miR-188-3p among mammals by Targetscan (Targetscan Human 7.2 version released) and two potential binding sites (in red) were analyzed in 3′-UTR of TMED3. **c** Double Luciferase reporter assay was performed between miR-188-3p and 3′-UTR of TMED3 in MCF-7 cells. **p < 0.01 compared with control using independent sample T-test. **d** Likewise, Luciferase reporter assay was performed in parallel in MDA-MB-231 cells. **p < 0.01 compared with control using independent sample T-test. **e** Variation of TMED3 mRNA was detected by qRT-PCR after transfection with miR-188-3p mimics and inhibitor sequence in MCF-7 and MDA-MB-231 cells, *p < 0.05 compared with control group. Shown were the representative figures selected among independent three times of repeats. **f**, **g** Variation of TMED3 on protein level was evaluated by western-blot, presented was the representative figure picked out from three times of independent repeat. Densitometric analysis of TMED3 blots were performed using Image J software (NIH, Bethesda, USA). **h** Detection of miR-188-3p by qRT-PCR in breast cancer (BCa) tissues and its matched normal controls, totaling 37. U6, as internal loading control; ***p < 0.001 compared with normal control using independent sample T-test; **i** correlation between miR-188-3p and TMED3 expression level was analyzed using Pearson correlation test in 37 cases of BCa; r = − 0.6656, p < 0.001 using Pearson Correlation test

### MiR-188-3p prevents from proliferation, migration and invasion in MCF-7 cells

Observing that miR-188-3p was significantly reduced in breast cancer tissues, we postulate that miR-188-3p may be anti-oncogenic in breast cancer. To test our postulation, we constructed the lenti-viral based miR-188-3p over-expression and its blank control vectors, followed by transfection into MCF-7 and MDA-MB-231 cells. As stated before, to single out those cells failing to be transfected, all the cells were subjected to cell sorting using Flow Cytometry platform. After sorting, all the positive cells sorted out were expanded in vitro. Then, we evaluated the effect of miR-188-3p on migration and invasion of MCF-7 and MDA-MB-231 cells through Transwell assay. It can be seen that forced expression of miR-188-3p can remarkably impair the migration and invasion of MCF-7 and MDA-MB-231 (Fig. 5a, b). Result from clonogenesis assay showed that re-expression of miR-188-3p can significantly suppress the clonogenic ability of MCF-7 and MDA-MB-231cells (Fig. 5c). On the other hand, apoptotic analysis of MCF-7 also indirectly supports the growth-suppressing role that re-expression of miR-188-3p can substantially induce the apoptosis of MCF-7 and MDA-MB-231 cells (Fig. 5d). As verification, xenograft nude mice model was used. MCF-7 cell line whose miR-188-3p has been stably enhanced was subcutaneously injected with 1 × 10^7^ cells. It presented that the growth of MCF-7 cells were pronouncedly inhibited in vivo (Fig. 5e, f), demonstrative of the suppression of growth of miR-188-3p in breast cancer. Moreover, to further confirm the maintenance of re-expression of miR-188-3p in MCF-7 cells, both qRT-PCR and western-blot were performed to detect the expression of miR-188-3p and TMED3 (Fig. 5g, h), respectively in tumor lesions dissected from nude mice that euthanatized. It showed that re-expression of miR-188-3p can be maintained at the time of end point as designed.

**Fig. 5:** MiR-188-3p suppresses migration, invasion and proliferation in BCa cells. **a** miR-188-3p was shown to suppress the migration in MCF-7 and MDA-MB-231 cells, as evaluated by Transwell assay. **p < 0.01 compared with control sing independent sample T-test; scale bar, 200 μm. **b** Similarly, miR-188-3p was presented to inhibit the invasion of MCF-7 and MDA-MB-231 cells, as assayed by Transwell, too. **p < 0.01 compared with control using independent sample T-test. Scale bar, 200 μm. **c** miR-188-3p was displayed to significantly slow down the proliferation in MCF-7 and MDA-MB-231 cells using Clonogenic assay. ***p < 0.001 compared with control using independent sample T-test. Shown was representative figure picked out of three times of independent repeats; **d** miR-188-3p can pronouncedly induce the apoptosis in MCF-7 and MDA-MB-231 cells, as analyzed by Flow Cytometry. ***p < 0.001 compared with control group using independent sample T-test. **e** Xenograft nude mice model demonstrated that miR-188-3p can significantly inhibit the growth of MCF-7 cells in vivo. **f** Kinetic growth curve of tumor lesion were plotted. *W* week; **g** qRT-PCR detection of miR-188-3p expression level in tumor lesions dissected from xenograft nude mice, *p < 0.001 compared with control; **h** western-blot detection of variation of TMED3 in tumor lesions dissected. Shown was representative figure picked out of three times of independent repeats

## Discussion

In our present investigation, to the best of our knowledge, we firstly showed that compared to normal controls, TMED3 was markedly up-regulated in breast cancer; that elevated TMED3 significantly clinicopathologically correlated with ER, PR, HER-2 status, lymph nodes metastases and inferior overall prognosis; and that in vitro cell lines, TMED3 was shown to promote the proliferation, migration and invasion of breast cancer cells. Moreover, miR-188-3p was identified to negatively modulate the TMED3. All the data we collectively obtained are strongly suggestive of its oncogenic role in breast cancer. Our findings are important in that we firstly defined the oncogenic role of TMED3 in breast cancer.

TMED3, also aliased C15orf22 or P26, a contraction of Transmembrane Emp24 Protein Transport Domain Containing 3, whose potential role has been proposed to be implicated in vesicular protein trafficking [13], mainly in the early secretory pathway. Besides, its physiopathological role remains unknown owing to little study has been emerged regarding TMED3 in the tumor setting, with the exception of three relevant studies performed in prostate cancer [10], colon cancer [11] and liver cancer [12] in chronological order. Analysis of the three previous studies [10–12] is readily indicative of its contradictory roles involved in the malignant behaviors of cancer. Original study of TMED3 on tumor came from prostate cancer by Vainio et al. [10] reporting that TMED3 whose mRNA was shown to be highly expressed in prostate cancer and high mRNA of TMED3 significantly correlated with AR and ERG oncogene expression, indicating the oncogenic trait of TMED3 that could be used as potential drug target in prostate cancer. Subsequent study of TMED3 carried out in colon cancer by Duquet et al. [11], however, seems to conflict with it. Duquet et al. [11] employed subcutaneous xenograft model demonstrating that TMED3 turns out to be able to suppress the metastasis of colon cancer through positive modulation of WNT-TCF pathway, strongly suggesting the tumor-suppressing role in colon cancer. In stark contrast with the observation by Duquet et al., Zheng et al. reported that up-regulated TMED remarkably correlated with aggressive malignant behaviors and poor prognosis in patients with hepatocellular carcinoma and TMED3 was shown to promote cell migration and invasion through IL-11/STAT3 signaling pathway [12]. In our present study, in terms of expression level, our observation made in breast cancer tissues were fully consistent with what’s been earlier reported in hepatocellular carcinoma [12] and prostate cancer [10] where TMED3 was found to be significantly up-regulated in cancer tissues compared with its normal controls. In study of TMED3 on colon cancer by Duquet et al. [11], in spite of lots of mechanistic data from mice model and cell culture system, the authors failed to analyze the expression patter of TMED3 on clinical tissue level. Moreover, when it comes to correlation with unfavorable overall prognosis and aggressiveness of cancer, our data was totally supported by the study of TMED3 in hepatocellular carcinoma by Zheng et al. [12]. These discrepancies, whatever in vivo or in vitro, between our study and what has been previous reported regarding TMED3 could be explained by the tissue-specific expression of TMED3, which would be tempting to speculate that TMED3 would be higher in secretory gland tissues compared with other glands, including breast, salivary, pancreas, prostate, gallbladder and thyroid glands etc., mainly based on its proposed biological roles that involved in protein trafficking and secretion. The speculation certainly needs to be confirmed in the following.

Mechanistically, the limited evidence available suggests that TMED3 worked through positive modulation of WNT-TCF [11] and IL-11/STAT3 [12] signaling pathways in colon and hepatocellular carcinoma, respectively. Different from the two studies mentioned, we attempted to search out the potential miRNA regulating the TMED3 with the help of miRNA microarray. Five significantly differential miRNAs were eventually screened out. Following the literature review and analysis, miR-188-3p was picked out and identified as negative regulator of TMED3 in breast cancer, among the candidate miRNA available. Although several studies were performed concerning miR-188 in cancers that defined miR-188 as tumor suppressor, miR-188-3p has been little described in cancers, not to mention in breast cancer except from only one recent study performed in colorectal cancer [14]. it has to be mentioned that miR-188-5p, another paralog of miR-188-3p from the same miR-188, was chorally reported to be tumor suppressing in cancers, including gastric [15], prostatic [16] and hepatocellular [17] carcinoma. Yet, in colorectal cancer, miR-188-3p was turned out to be significantly elevated in cancer tissues relative to normal controls and re-expression of miR-188-3p was therefore shown to promote migration and invasion of colorectal cancer cells in vitro, indicating its oncogenic property in colorectal cancer. By contrast, in our study, miR-188-3p was found to be markedly down-regulated in breast cancer compared with its normal control. In vitro functional analysis of miR-188-3p supported the tumor suppressing role in breast cancer cells, taking the form of suppression of proliferation, migration and invasion in MCF-7 cells. As further verification, Pearson correlation analysis on tissue level corroborated the luciferase reporter assay performed in vitro breast cancer cell lines, confirming the negative modulation of miR-188-3p on TMED3.

## Conclusion

Collectively, we firstly defined the oncogenic role of TMED3 in breast cancer showing that elevated TMED3 significantly correlated with inferior overall prognosis as well as ER, PR and HER2 status and that TMED3 can promote proliferation, migration and invasion of breast cancer cells in vitro. Furthermore, miR-188-3p can negatively regulate TMED3, suppressing the proliferation, migration and invasion of breast cancer cells in vitro.

## Additional file

**Additional file 1: Figure S1.** TMED2, TMED3 and TMED4 expression in breast cancer cell lines. **A**: qRT-PCR detection of TEMD2, TMED3 and TMED4 in a plethora of breast cancer cell lines; **B**: qRT-PCR detection of TEMD2, TMED3 and TMED4 in MCF-7 and MDA-MB-231 cells we used. *p < 0.05 compared with MCF-7 group, acting as control; C: western-blot detection of TEMD2, TMED3 and TMED4 in MCF-7 and MDA-MB-231 cells we used. The molecular weight of TMED2, TMED3 and TMED4 was observed to be 23 kDa, 25 kDa and 26 kDa, respectively; β-Tubulin, internal loading control, whose molecular weight was observed to be around 55 kDa. **Figure S2.** TMED3 prevents apoptosis and increases S phase in breast cancer cell lines. A: stable silencing of TMED3 was found to pronouncedly induce the earlier apoptosis in MCF-7 and MDA-MB-231 cell lines, as shown by Flow Cytometry analysis; ***p < 0.001 in comparison with control group using independent sample T-test; B: Meanwhile, MCF-7 and MDA-MB-231 cells subjected to apoptotic analysis were in parallel subjected to cell cycle analysis. Stable knock-down of TMED3 was able to decrease percent of the S phase while increasing G1 phase. All flow cytometric assays were carried out independently three times and shown were representative figures picked out among candidates. **Figure S3.** Bioinformatic analysis of binding site of miR-188-3p in 3′-UTR sequence of TMED3. Highlighted site means binding sites of miR-188-3p.
